This article has been retracted.

# Repertoire of the gut microbiota from stomach to colon using culturomics and next-generation sequencing

**DOI:** 10.1186/s12866-018-1304-7

**Published:** 2018-10-24

**Authors:** Morgane Mailhe, Davide Ricaboni, Véronique Vitton, Jean-Michel Gonzalez, Dipankar Bachar, Grégory Dubourg, Frédéric Cadoret, Catherine Robert, Jérémy Delerce, Anthony Levasseur, Pierre-Edouard Fournier, Emmanouil Angelakis, Jean-Christophe Lagier, Didier Raoult

**Affiliations:** 1 Aix Marseille Univ, IRD, MEPHI, IHU - Méditerranée Infection, 19-21 Boulevard Jean Moulin, 13005 Marseille, France; 2 Department of Clinical and Biomedical Sciences Luigi Sacco, III Division of Infectious Diseases, University of Milano, Via GB Grassi, 74, 20157 Milan, Italy; 3 Service de Gastroentérologie, Hôpital Nord, Assistance Publique-Hôpitaux de Marseille, 13915 Marseille, France; 4 Aix Marseille Univ, IRD, VITROME, IHU - Méditerranée Infection, 19-21 Boulevard Jean Moulin, 13005 Marseillle, France

**Keywords:** Gut microbiota, Culturomics, Metagenomics, New species

## Abstract

**Background:**

Most studies on the human microbiota have analyzed stool samples, although a large proportion of the absorption of nutrients takes place in upper gut tract. We collected samples from different locations along the entire gastrointestinal tract from six patients who had simultaneously undergone upper endoscopy and colonoscopy, to perform a comprehensive analysis using culturomics with matrix assisted laser desorption ionisation - time of flight (MALDI-TOF) identification and by metagenomics targeting the 16S ribosomal ribonucleic acid (rRNA) gene.

**Results:**

Using culturomics, we isolated 368 different bacterial species, including 37 new species. Fewer species were isolated in the upper gut: 110 in the stomach and 106 in the duodenum, while 235 were isolated from the left colon (*p* < 0.02). We isolated fewer aero-intolerant species in the upper gut: 37 from the stomach and 150 from the left colon (*p* < 0.004). Using metagenomics, 1,021 species were identified. The upper gut microbiota was revealed to be less rich than the lower gut microbiota, with 37,622 reads from the stomach, 28,390 from the duodenum, and 79,047 from the left colon (*p* < 0.009). There were fewer reads for aero-intolerant species in the upper gut (8,656 in the stomach, 5,188 in the duodenum and 72,262 in the left colon, *p* < 0.02).

Patients taking proton pump inhibitors (PPI) were then revealed to have a higher stomach pH and a greater diversity of species in the upper digestive tract than patients not receiving treatment (*p* < 0.001).

**Conclusion:**

Significant modifications in bacterial composition and diversity exist throughout the gastrointestinal tract. We suggest that the upper gut may be key to understanding the relationship between the gut microbiota and health.

**Electronic supplementary material:**

The online version of this article (10.1186/s12866-018-1304-7) contains supplementary material, which is available to authorized users.

## Background

The gut microbiota plays an important part in harvesting, storing and expending energy obtained from the diet. Previous studies have shown that the absorption of fat, simple carbohydrates and proteins begins in the duodenum and is completed in the jejunum [1]. The distal part of the small intestine is mainly involved in the absorption of bile acids and vitamin B12, while the colon is responsible for the absorption of water, electrolytes and short chain fatty acids produced by bacterial fermentation [2]. Overall, the colon receives only 15% of ingested carbohydrates and 5–33% of proteins [3]. Microbiota taxonomic complexity and bacterial load increases gradually from the stomach (10^1^–10^3^ CFU/ml) to the jejunum (10^4^–10^7^ CFU/ml) to feces (10^11^–10^12^ CFU/ml) [4, 5], which mainly consists of aero-intolerant prokaryotes [6]. In the small intestine, the transit time is short, and the presence of digestive enzymes and bile makes the environment inhospitable to microbial life. There, the resident microbiota exhibits less species diversity but greater inter-subject variability compared to the mouth or colon [7]. The gut microbiota of the small intestine is dominated by *Streptococci*, *Bifidobacterium*, *Enterococci* and *Lactobacilli* which successfully develop metabolic pathways centered on the rapid uptake and conversion of simple carbohydrates [8]. Studies linking obesity and the gut microbiota focus on differential small intestine bacterial efficiency in carbohydrates and fatty acid oxidation, with the consequent Cholecystokinin-mediated feedback on the satiety reflex [9], whereas the presence of *Lactococcus sp.* in this part of the intestine has been associated with the lipid and carbohydrate metabolisms [10].

The composition of the human gut microbiota was significantly revived by metagenomic studies. However, 16S rRNA sequencing-based methods are biased by the different deoxyribonucleic acid (DNA) extraction methods used [11] and can lead to an overestimation of bacterial proportions. In addition, culturomics consists of the application of high-throughput culture conditions to the study of the human microbiota and uses MALDI-TOF or 16S rRNA amplification and sequencing for identifying growing colonies, some of which have been previously unidentified [12]. Culturomics, a high throughput culture method with rapid identification by MALDI-TOF has proven to be highly complementary with metagenomics [13], with an overlap of only 15% of detected species when applied to the same samples [14]. Successive studies have confirmed the complementarity of these two techniques [15, 16].

We believe that the human-gut functional subdivision corresponds an equally specific microbiota functional compartmentalization that is missed when working exclusively on fecal samples. To date, few human gut microbiota studies have involved samples from the entire gut tract, in comparison to studies using stool samples [17]. To reach our goal of getting the most complete panorama of the entire gut host microbiota relationship [18], during the same endoscopy session, we collected samples from five different locations along the entire gastrointestinal tract. All the samples were subjected to high-throughput 16S rRNA gene amplicon sequencing and culturomics.

## Results

### Physicochemical characteristics of the samples

The physicochemical characteristics of all samples were measured (Additional file 1**:** Table S2). The mean ± SD pH was significantly lower in the stomach and duodenal samples for untreated patients compared to patients receiving PPI (1.8 vs 7.0 and 2.5 vs 7.1, *p* < 0.001 respectively) (Fig. 1). No difference was found between these two groups for samples from the ileum, right and left colon (Additional file 2: Figure S1).

**Fig. 1:** Comparison of digestive levels according to whether or not patients were treated with PPIs. As no normalization has been performed before PCR reaction, no significant conclusion can be supported regarding the density of the bacteria, the number of reads is indicated with informative value. *Firmicutes*: blue, *Proteobacteria*: red, *Bacteroidetes*: green, *Actinobacteria*: yellow, *Fusobacteria*: pink. Ai: aerointolerant, Ae: aerotolerant

### Culturomics

A total of 26,128 colonies were tested by MALDI-TOF MS with a mean ± SD of 4,355 ± 797 (ranging from 3,268 to 5,304) per patient and 368 different bacterial species were identified (Additional file 3**:** Figure S2). In total, 219 (60%) isolates were strictly aero-intolerant. The bacterial species belonged to *Firmicutes* (*n* = 193 different species, 52%), followed by *Bacteroidetes* (*n* = 68, 18%), *Actinobacteria* (*n* = 61, 17%), *Proteobacteria* (*n* = 36, 10%), *Fusobacteria* (n = 6, 2%), *Synergistetes* (*n* = 2, 0.4%), *Verrucomicrobia* (n = 1, 0.2%) and *Lentisphaerae* (n = 1, 0.2%) (Additional file 4**:** Table S3). These isolates belonged to 141 different genera: *Clostridium* was the most common (*n* = 24, 7%) followed by *Bacteroides* (*n* = 21, 6%)*, Streptococcus* (n = 21, 6%) and *Lactobacillus* (*n* = 16, 4%). In total, 304 (83%) bacterial species were bacteria previously described in the human gut (Fig. 2a), whereas 23 (6%) species were bacteria already described in human other site but not in the gut and were isolated for the first time in the human gut in this study, 4 (1%) were known species from the environment but were isolated for the first time in humans, and 37 (10%) were new bacterial species isolated for the first time (Additional file 5: Table S4) of which we identified 17 new genera. All these new prokaryote species have undergone whole genome sequencing and described using the taxonogenomic approach [19–21]. They have been deposited in a strain collection: the Collection de Souches de l’Unité des Rickettsies (CSUR).

**Fig. 2:** **a**) Species isolated by culturomics along the digestive tract in terms of whether they are known in the gut (green), in humans (yellow), in the environment (orange), and or whether they have been isolated for the first time (red). **b)** Venn diagram representing bacterial species numbers identified by culturomics (green) and metagenomics (red), with the percentage of species found by both approaches, for each patient and each step along the digestive tract

We looked for the presence of a bacterial core on the basis of culturomics but we did identify any common bacterial species in all samples tested. However, eight different species (*Bacteroides ovatus*, *Bacteroides uniformis*, *Bacteroides vulgatus*, *Bifidobacterium longum*, *Clostridium lavalense*, *Escherichia coli*, *Flavonifractor plautii* and *Streptococcus mitis*) were isolated in at least 50% of the samples tested.

### Metagenomics

Metagenomics enabled the identification of 16 different bacterial phyla (Additional file 3**:** Figure S2). Most of the Operational Taxonomic Unit (OTUs) assigned to known species belonged to *Firmicutes* (*n* = 418, 41%), followed by *Proteobacteria* (*n* = 294, 29%), *Bacteroidetes* (*n* = 134, 13%), *Actinobacteria* (n = 134, 13%), *Fusobacteria* (*n* = 11, 1%), *Spirochaetes* (*n* = 6, 0.6%), Synergistetes (*n* = 5, 0.5%), *Verrucomicrobia* (*n* = 3, 0.3%), *Cyanobacteria* (n = 3, 0.3%), *Deinococcus-Thermus* (n = 3, 0.3%), *Tenericutes* (n = 3, 0.3%), *Acidobacteria* (n = 2, 0.2%), *Aquificae* (n = 3, 0.3%), *Lentisphaerae* (n = 1, 0.1%), *Negibacteria* (n = 1, 0.1%) and *Saccharibacteria* (n = 1, 0.1%) (Additional file 4**:** Table S3). Throughout the study 1,021 bacterial species were identified by this approach (Additional file 6**:** Figure S3), with a mean value of 434 ± 75 species per patient (ranging from 315 to 518). In particular, *Methanobrevibacter smithii* was identified in the ileum, right and left colon of patient 1 and in the stomach and left colon of patient 3.

The existence of a common bacterial core among the different parts of the digestive tract was then examined. We found that five different genera (*Bacteroides*, *Blautia*, *Escherichia*, *Lachnoclostridium* and *Streptococcus*) and three different species (*Bacteroides uniformis*, *Escherichia coli* and *Streptococcus salivarius*) were detected in all the samples. Moreover, we found 64 (6%) different genera and 103 (10%) different species in at least 50% of the samples tested.

### Comparison between culturomics and metagenomics

Overall, 1,195 known species were identified: 174 (15%) were only identified by culturomics, 827 (69%) only by metagenomics, and 194 (16%) species by both (Fig. 2b).

Significantly the proportion of aero-intolerant species was found to be higher using culturomics (219, 60%) than metagenomics (430, 42%) (*p* < 0.001).

In addition, we used blast to compare the 16S rRNA sequences of the 37 new species isolated by culturomics with the non-identified OTUs from the 16S rRNA of all samples (Additional file 5**:** Table S4). All these species were also detected by metagenomics, corresponding to 11,990 reads (Fig. 3).

**Fig. 3:** Principal component analysis conducted on all samples, showing the difference between upper and lower parts of the digestive tract

### Comparison of the different parts of the digestive tract

Using culturomics, no differences were found between the number of species isolated in the stomach (*n* = 110, 30%) compared to the duodenum (*n* = 106, 29%) but significantly fewer when compared to the ileum (*n* = 185, 50% with *p* = 0.02), and the right and left colon (*n* = 200, 54% and *n* = 235, 64% with *p* = 0.009 respectively) (Additional file 6**:** Figure S3a). In addition, we found significantly fewer aero-intolerant species in the stomach (*n* = 37, 34%) and duodenum (*n* = 46, 43%) than in the ileum (*n* = 116, 63% with *p* = 0.004), and the right and left colon (*n* = 137, 69% and *n* = 150, 64% with *p* = 0.002 respectively) (Additional file 6**:** Figure S3b).

Metagenomics revealed significantly fewer reads in the stomach (n = 37,622, 14%, with *p* = 0.009) and the duodenum (*n* = 28,390, 10%, with *p* = 0.004) than in the left colon (*n* = 79,047, 29%) (Additional file 6**:** Figure S3d). The microbiota of the stomach and the duodenum presented significant less richness (estimated by the Chao1 index) and biodiversity (assessed by a nonparametric Shannon index) than the ileum (*p* = 0.009 and *p* = 0.01 respectively), the right (*p* = 0.007 and *p* = 0.009 respectively) and the left colon (*p* = 0.004 and *p* = 0.007 respectively) (Additional file 7**:** Figure S4). In addition, we observed significantly fewer reads for aero-intolerant species in the stomach (*n* = 8,656, 23%) and the duodenum (*n* = 5,188, 18%) than in the ileum (*n* = 62,356, 89%) (*p* = 0.02 each), right colon (*n* = 52,499, 90%, with *p* = 0.0004 and *p* = 0.0001 respectively) and left colon (*n* = 72,262, 91%, with *p* = 0.004 and *p* = 0.003 respectively) (Additional file 6**:** Figure S3e). It is interesting to note that some phyla were identified only in the upper gastrointestinal tract and not in the lower digestive tract such as *Spirochaetes*, *Deinococcus-Thermus*, *Tenericutes*, *Acidobacteria*, *Aquificae* and *Negibacteria* (Additional file 4**:** Table S3).

Principal component analysis (PCA) revealed a relationship between the stomach microbiota and low pH (Fig. 4). Stomach samples were clustered with more *Proteobacteria* and fewer *Firmicutes* or *Bacteroidetes*. The duodenum was associated with a lower index of Shannon highlighting the diversity and a lower number of reads as previously described by other methods [22]. At this anatomical level, there were more *Actinobacteria* and fewer *Firmicutes*. Moreover, this upper part of the digestive tract was associated with a predominance of aerotolerant species. In contrast, there was a predominance of strict aero-intolerant species in the right and left colon. The ileum and right and left colons were associated with the presence of *Firmicutes* and *Bacteroidetes.* These parts also clustered with a higher pH and Shannon index, species and read numbers.

**Fig. 4:** Neighbor-joining phylogenetic with the non assigned OTUs from the 16S rRNA of all samples corresponding to the 37 new species identified in culturomics in red

### Comparison of the gut of patients receiving treatment with PPIs to those who were not

We observed a significant relationship between taking PPIs and a higher pH. This was confirmed by PCA, as well as the Shannon index and the number of different species. In the untreated group, we isolated 754 species, including 377 aero-intolerant species (50%) and in the group treated with PPIs, we identified 960 species including 462 aero-intolerant species (48%) using the two techniques. Patients taking PPIs had a greater diversity of bacterial species than patients not receiving treatment (*p* < 0.001). Patients treated with PPIs had a higher recovery percentage revealed by both techniques than the untreated group (Fig. 2b). There was no difference in the metabolism of these species in the two groups.

No significant differences were found between phyla distribution in the two groups in any part of the digestive tract.

## Discussion

To the best of our knowledge, this work is the first comprehensive analysis combining metagenomics and culturomics, performed using staged specimens of the human gut. We analyzed samples from five different locations along the entire gastrointestinal tract and revealed that the human microbiota presents significant changes. All analyzed samples were collected under similar conditions, were freshly inoculated to promote the growth of aero-intolerant bacterial species and were frozen under sterile conditions at − 80 °C, eliminating the possibility of contamination. We concomitantly used two DNA extraction protocols to observe the greater diversity, as previously described [13]. In addition, the V3-V4 region was targeted for 16S rRNA sequencing, as widely used in the literature for determination of the gut microbiota [23]. Moreover, for culturomics, which has previously demonstrated its efficiency in terms of increasing the gut microbiota repertoire, we selected the most profitable culture conditions, analyzing former studies on this topic [5, 14]. We used negative controls to test the veracity of our results. However, one limitation of our study was that, due the difficulty of performing upper endoscopies and colonoscopies, we did not use samples from healthy volunteers for this study, but from patients with various diseases, including one with Crohn’s disease. We observed a difference in the microbiota composition of the patient with Crohn’s disease with respect of the other patients but we could not conclude because of the small number of patients. This patient had a less richness microbiota than the other five. By culturomics, we isolated only 63 different species in the patient with Crohn’s disease while an average of 132 species were isolated from the other five. By metagenomics, we identified only 315 different species in the patient with Crohn’s disease (with 39% of anaerobes) while an average of 597 species were isolated from the other five (with 59% of anaerobes). Moreover, the consequence of the significant workload, notably for culturomics studies, is that only a small number of patients were tested. Among the biases of our study, besides even if the maximum of precaution was taken during the endoscopic examination, a possible contamination remains possible of a site with high density at a site with less density in bacteria. However, this is unlikely because of differences in concentration and composition detected in the different samples.

We observed a dramatic divergence between the sets of bacteria identified by culturomics and metagenomics at both species and genera level. Indeed, only 194 bacterial species were common between the two approaches, while 174 species were only detected by culturomics. Our results confirm previous studies, which also revealed an important complementarity between these two techniques [14–16]. Characterized by their depth bias, metagenomic methods are unable to detect small populations of prokaryotes [24]. Nevertheless, several taxa have been detected in human beings using this technology. Moreover, we isolated 37 new species: the sequences of all these species were retrieved by metagenomics, but their absence from the National Center for Biotechnology Information (NCBI) database meant that some OTUs were not assigned to a known species. Consequently, this work again contributes towards shedding light on part of bacterial dark matter [12, 25]. All of them will be comprehensively described using taxonogenomics [19–21].

We observed an increasing gradient in the number of reads and the number of isolates when comparing the upper gastrointestinal tract with the lower. The increasing degree of bacterial diversity along the gut had already been previously reported. The acidic environment in the stomach, the oxygen gradient from the mouth to the rectum, the transit speed, the biliary salts, the mucosal secretion of IgA, and the secretion of antimicrobials by Paneth cells in the small intestine may explain the lower bacterial diversity in the upper gastrointestinal parts [26, 27]. In addition, the upper digestive tract was colonized by aerotolerant bacteria, while there was a significant predominance of aero-intolerant species in the right and left colon. Indeed, *Proteobacteria* were significantly more common in the upper part of the gut, while *Bacteroidetes* were significantly more common in the lower tract [28]. Previous studies described the existence of an oxygen gradient from the relatively oxygenated colonic submucosa to the more anoxic lumen [29], with special attention being paid to the consequences of this gradient on the distribution of the microbiota [30]. Other studies have reported the existence of another decreasing oxygen gradient from the mouth to the rectum with PaO_2_ (mmHg) of 46.3 ± 15.4 in the stomach compared to 29.3 ± 11 in the colon [31, 32]. To our knowledge, this is the first study focusing on the evolution of the microbiota from the stomach to the left colon according to oxygen tolerance.

Our results are astonishing compared to the literature [33] but we found a gastric pH at 7 after taking PPIs. Our method was the same regardless of whether patients had PPIs or not. The small amount of sterile saline solution was injected during the endoscope progression whether the patients were under PPI or not. This method did not change the pH of the samples because we can observe that pH of the high digestive tract samples without PPI was around 2 with this same method. Moreover, PPI treatment results in modifications in the gut microbiota, with an increase in the *Firmicutes* population associated with a decrease in *Bacteroidetes*. Similarly, previous studies have revealed important microbiota changes in the terminal ileum with PPI administration, which can be summarized as an increase in *Firmicutes* (*Lactobacillus* or *Clostridium*) and/or a decrease in *Bacteroidetes* [34, 35]. Furthermore, alterations in the gut microbiota (a decrease in *Akkermansia* and *Coprococcus* and an increase in *Bacteroidales*) and weight loss after the administration of omeprazole in C57BL/6 J mice has been reported [36]. Moreover, we observed that patients treated with PPIs presented increased gut flora diversity. In contrast, in two previous studies it was found that the use of PPIs is associated with lower diversity [37, 38], while yet another study revealed no impact of PPI use on overall bacterial diversity [35]. PPI use is associated with weight loss [39], but this may depend upon an individual’s underlying obesity or gut microbiota [40, 41].

## Conclusion

This work revealed that the gut microbiota is much different from its upper part, where foods are absorbed, and its lower part, the colon, which can be likened to waste, with bacterial growth due to fermentation [42]. This exhaustive analysis of the digestive microbiota of tiered samples will make it possible to compare healthy and diseased populations, such as obese patients, cirrhotic patients, and even patients with cancer [43].

## Methods

### Patients and samples

We used samples from the stomach, duodenum, ileum, right and left colon from patients who had simultaneously undergone an upper endoscopy and colonoscopy for diagnostic purpose between February and June 2016 at the Hôpital Nord (Aix-Marseille University, AP-HM, Gastro-enterology Department, Hôpital Nord, Marseille, France). Patients were excluded if, in the previous 6 months, they had received antibiotherapy or had taken a trip outside Europe. Patients gave their signed informed consent and completed a clinical questionnaire. Overall, six adult volunteers (three males, three females) were include (Table 1) with a mean ± standard deviation (SD) age of 49 ± 18 and mean ± SD body mass index of 26.5 ± 7 kg/m^2^. They included one obese patient (patient 3) and one patient with a Crohn’s disease (patient 4). Three patients were currently receiving long-term treatment with PPI: patient 1 because of a gastro-esophageal reflux, patient 2 because of a gastric ulcer and patient 6 because of an esophagitis (Table 1). The ethics committee of the Institut Hospitalo-Universitaire (IHU) Méditerranée Infection validated the study under number 2016–010.

**Table 1:** Patients’ characteristics of our study

Patient	Age (years)	BMI (kg/m^2^)	Diseases	Diet	PPI
1	51–60	24.3	Gastro-esophageal reflux	no	yes
2	51–60	21.5	Gastric ulcer	no	yes
3	21–30	41.8	Obesity	no	no
4	21–30	21.3	Crohn’s disease	residue-free	no
5	41–50	24.2	Flatulence	no	no
6	71–80	26	Esophagitis	probiotics	yes

*BMI* body mass index, *PPI* proton pump inhibitor

All samples were taken during gastroscopy and colonoscopy by injection and the prompt aspiration of sterile saline solution. To preserve extremely oxygen sensitive strains, samples destined for liquid enrichment were immediately inoculated after collection, in a blood culture bottle (BD BACTEC®, Plus Anaerobic / F Media, Le Pont de Claix, France) previously supplemented with 5 ml of sheep blood and 5 ml of 0.2 μm filtered rumen [6]. Samples destined for direct plating on solid agar media were placed in antioxidant transport medium immediately after collection [44] and seeded within 2 hours. Once in sterile conditions in the laboratory, the fresh samples were aliquoted, and a part was stored at − 80 °C for metagenomic study. The redox potential, pH and salinity were measured from all the samples, as previously described [45].

### Culturomics

All samples were cultured in eight different agar media (Additional file 8: Table S1) as previously described [13]. In addition, for samples from the stomach, duodenum and ileum, culturing was performed on a ninth medium and for the right and left colon samples, a heat shock (20 min at 80 °C) was also performed before inoculation on Columbia agar with sheep blood (Columbia agar + 5% sheep blood, bioMérieux, Marcy l’Etoile, France). To perform direct seeding, the fresh samples were serially diluted with 0.1 M PBS (Dulbecco’s Phosphate-Buffered Saline, ThermoFisher Scientific, Paisley, UK) and immediately spread on the different culture media. All Petri dishes were incubated at 37 °C and were subcultured under the same conditions after 3, 7 and 10 days. For the samples that underwent liquid enrichment, plating and subcultures were performed on 5% sheep blood agar (bioMérieux) under anaerobic conditions on days 1, 3, 7, 10, 15, 21 and 30.

### MALDI-TOF mass spectrometry

As previously described, the bacterial isolates were identified using MALDI-TOF mass spectrometry (MALDI-TOF MS, Bruker Daltonics, Billerica, Mass., USA) to quickly identify the colonies [46]. Each isolate was deposited on a MALDI-TOF target in two spots and covered with a matrix solution (α-cyano acid 4-hydroxycinnamic acid diluted in 500 μl of acetonitrile, 250 ml of acid tri-fluoro-acetic acid in 10% water and 250 ml of HPLC). Automatic acquisition of the spectra was performed using FlexControl 3.0 software, and analysis was performed using the Biotyper 2.0 software. An isolate was considered to have been correctly identified at the species level when at least one spectrum had a score ≥ 1.9. For the unidentified isolates, polymerase chain reaction (PCR) amplification and sequencing of the 16S rRNA gene was performed [47].

### Molecular assays

Total genomic DNA was extracted from colonies using a QIAamp tissue kit (Qiagen, Hilden, Germany) and stored at 4 °C until use for PCR amplification and sequencing of the 16S rRNA gene, using previously described methods [48]. All sequences were compared with those available in the GenBank, European Molecular Biology Laboratory (EMBL) and Daniel J. Bernstein (DJB) databases using the gapped BLASTN 2.0.5 program through the National Center for Biotechnology Information server. A threshold similarity of > 98.7% was chosen to define a new bacterial species [49].

### Extraction of DNA from samples and 16S rRNA sequencing using MiSeQ technology

Thirty samples were extracted from six patients in both protocols as previously described in the literature. This concomitant extraction by two protocols (named protocol 1 and protocol 5) including one protocol with a deglycosylation step [50]. Indeed, we performed the amplification of 60 samples, which were barcoded, pooled and then sequenced for 16S rRNA sequencing on MiSeq technology (Illumina, Inc., San Diego CA 92121, USA) using the paired-end strategy constructed according to the 16S Metagenomic Sequencing Library Preparation (Illumina). For 16S rRNA sequencing, DNA was amplified for the 16S “V3-V4” regions by PCR, using the Kapa HiFi Hotstart Ready Mix (Kapabiosystems, Wilmington, MA USA) and the surrounding conserved region V3_V4 primers with overhang adapters (FwOvAd_341F TCGTCGGCAGCGTCAGATGTGTATAAGAGACAGCCTACGGGNGGCWGCAG;RevOvAd_785RGTCTCGTGGGCTCGGAGATGTGTATAAGAGACAGGACTACHVGGGTATCTAATCC). After purification on AMPure beads (Beckman Coulter Inc., Fullerton, CA, USA), the concentration was measured using high sensitivity Qubit technology (Thermo Fisher Scientific Inc., Waltham, MA USA) and dilution to 3.5 ng/μl was performed. Using a subsequent limited cycle PCR on 52.5 ng of the cleaned PCR product, Illumina sequencing adapters and dual-index barcodes were added to the amplicon. After purification on AMPure beads (Beckman Coulter Inc., Fullerton, CA, USA), each library was pooled with other multiplexed samples and the concentration of this pool was re-measured using the Qubit® dsDNA HS Assay Kit and adjusted at 4 nM. Dilution at 4 pM was performed to load on the flowcell. Automated cluster generation and paired-end sequencing with dual index reads was performed in a single 39-h run in a 2 × 251 bp. A total of 4.1 Gb of information was obtained from a 439 K/mm^2^ cluster density with a cluster passing quality control filters of 94.8% (8,080,000 clusters). The raw data were configured in fastq files for R1 and R2 reads.

### Data processing: Filtering the reads, dereplication and clustering

The paired end sequences of corresponding raw fastq files were assembled into longer joined sequences by FLASH [51] with a quality score cut-off value of 33. Low quality reads were filtered out with QIIME [52]. Both the primers were removed from the sequences. Shorter (< 200 nts) and longer (> 1,000 nts) sequences were also discarded. Chimeric sequences were removed using Chimeraslayer [52]. De novo operational taxonomic unit (OTU) clustering of these sequences was performed using UCLUST [53] at 97% identity. The raw sequences of paired end reads in the fastq files were submitted to European Bioinformatics Institute (EMBL-EBI, http://www.ebi.ac.uk/).

### Building the reference database

From the Silva website, the Silva small and large subunit (SSU and LSU) database [54] of release 119 was downloaded. Then we extracted the Silva reference sequences containing both the forward and reverse primers, three differences between each primer and the sequence were allowed [55] to build a local database of predicted amplicon sequences.

Finally, our local reference database was used, containing a total of 456,714 well-annotated sequences.

### Taxonomic assignments

Blast were then used to search the OTUs against the Silva reference database [56]. The best matches ≥97% identity and 100% coverage for each of the OTUs was extracted from the reference database, and taxonomy was assigned up to the species level.

### Database of obligate aero-intolerant species

A bacterial oxygen tolerance database was set up based on the literature (available online at http://www.mediterranee-infection.com/article.php?laref=374). According to oxygen tolerance, each phylotype was assigned as ‘aero-intolerant’ or ‘aerotolerant’.

### Statistical analysis

With the mothur software package [57], we calculated the richness and biodiversity index of the OTUs. We used the Chao1 index to estimated richness and the non-parametric Shannon formula to estimated diversity [23]. We used the normalized option of Lefse for the linear discriminant [24] and QIIME for rarefaction and principal coordinate analysis [52]. A t-test was performed using Graph pad software and a principal component analysis was performed with Xlstat software. Statistical Package for the Social Sciences (IBM Corp. Released 2011. IBM SPSS Statistics for Windows, Version 20.0. Armonk, NY: IBM Corp.) was used to perform other statistical analyses.

## Additional files

Additional file 1: **Table S2.** Physicochemical characteristics of patient samples along the digestive tract. (DOCX 13 kb)

Additional file 2: **Figure S1.** Comparison of the pH samples along the digestive tract. (JPG 74 kb)

Additional file 3: **Figure S2.** Phyla identified along the gastrointestinal tract by culturomics (number of identified species): *Proteobacteria* (a), *Bacteroidetes* (b), *Firmicutes* (c) and metagenomics (number of generated reads): *Proteobacteria* (d), *Bacteroidetes* (e), *Firmicutes* (f), * *p* < 0.05. (TIFF 184 kb)

Additional file 4: **Table S3.** Number of species, ranged by phyla, along the digestive tract identified by culturomics, metagenomics and both assays. (DOCX 15 kb)

Additional file 5: **Table S4.** New bacterial species isolates by culturomics. (DOCX 19 kb)

Additional file 6: **Figure S3.** Number of identified species by culturomics (a), with aerointolerant (b) and aerotolerant (c) species identified along the digestive tract, and number of generated reads by metagenomics (d) with number of reads from aerointolerant (e) and aerotolerant species (f) along the digestive tract, * *p* < 0.05. (TIFF 197 kb)

Additional file 7: **Figure S4.** Shannon index along the digestive tract, * *p* < 0.05. (TIFF 62 kb)

Additional file 8: **Table S1.** Culture conditions used for culturomics in this study. (DOCX 13 kb)

## Abbreviations

AP-HM: Assistance Publique Hôpitaux de Marseille
CSUR: Collection de Souches de l’Unité des Rickettsies
DJB database: Daniel J. Bernstein database
DNA: Deoxyribonucleic acid
EMBL-EBI: European Molecular Biology Laboratory – European Bioinformatics Institute
IHU: Institut Hospitalo-Universitaire
LSU: Large subunit
MALDI – TOF MS: Matrix assisted laser desorption ionisation - time of flight mass spectrometry
NCBI: National Center for Biotechnology Information
OTU: Operational taxonomic unit
PBS: Phosphate-buffered saline
PCA: Principal component analysis
PCR: Polymerase chain reaction
PPI: Proton pomp inhibitors
rRNA: Ribosomal ribonucleic acid
SD: Standard deviation
SPSS: Satistical package for the social sciences
SSU: Small subunit
